The article "Effects of a Single Dose of Ivermectin on Viral and Clinical Outcomes in Asymptomatic SARS-CoV-2 Infected Subjects: A Pilot Clinical Trial in Lebanon" was retracted in 2021. Reason: errors in the analysis.

# Effects of a Single Dose of Ivermectin on Viral and Clinical Outcomes in Asymptomatic SARS-CoV-2 Infected Subjects: A Pilot Clinical Trial in Lebanon

**DOI:** 10.3390/v13060989

**Published:** 2021-05-26

**Authors:** Ali A. Samaha, Hussein Mouawia, Mirna Fawaz, Hamad Hassan, Ali Salami, Ali Al Bazzal, Hamid Bou Saab, Mohamed Al-Wakeel, Ahmad Alsaabi, Mohamad Chouman, Mahmoud Al Moussawi, Hassan Ayoub, Ali Raad, Ola Hajjeh, Ali H. Eid, Houssam Raad

**Affiliations:** 1 Faculty of Public Health, Lebanese University, Beirut, Lebanon; ali.samaha@liu.edu.lb (A.A.S.); houssein.mouawia@ul.edu.lb (H.M.); hamad.hassan@ul.edu.lb (H.H.); ali.albazzal@gmail.com (A.A.B.); doctorchouman@gmail.com (M.C.); dr.raad.ali@hotmail.com (A.R.); hajjehpharmacy@hotmail.com (O.H.); 2 Nursing Department, Faculty of Health Sciences, Beirut Arab University, Beirut, Mazraa 1105, Lebanon; mirna.fawaz@bau.edu.lb; 3 Department of Biomedical Sciences, Lebanese International University, Beirut, Mazraa 1105, Lebanon; 4 Department of Cardiology, Rayak University Hospital, Bekaa 1801, Lebanon; ayoub_hassan@yahoo.com; 5 Ministry of Health, Beirut, Lebanon; 6 Department of Mathematics, Faculty of Sciences, Lebanese University, Nabatieh 1700, Lebanon; a.salami@ul.edu.lb; 7 Faculty of Sciences, Lebanese University, Zahle 1801, Lebanon; h.bousab@ul.edu.lb; 8 Karbala Health Directory, Baghdad 10081, Iraq; mohammed.alwakeel1983@gmail.com; 9 Department of Biology, Lille University, 59160 Lille, France; ahmad_alsaabi@hotmail.com; 10 Faculty of Nursing Sciences, Islamic University of Lebanon, Baalbek 1800, Lebanon; dr.Mmouss@yahoo.com; 11 Department of Basic Medical Sciences, College of Medicine, QU Health, Qatar University, Doha, Qatar; 12 Biomedical and Pharmaceutical Unit, QU Health, Qatar University, Doha, Qatar

**Keywords:** ivermectin, SARS-CoV-2, COVID-19, Lebanon, clinical trial, pandemic, therapy

## Abstract

Objective: This study was designed to determine the efficacy of ivermectin, an FDA-approved drug, in producing clinical benefits and decreasing the viral load of SARS-CoV-2 among asymptomatic subjects that tested positive for this virus in Lebanon. Methods: A randomized controlled trial was conducted in 100 asymptomatic Lebanese subjects that have tested positive for SARS-CoV2. Fifty patients received standard preventive treatment, mainly supplements, and the experimental group received a single dose (according to body weight) of ivermectin, in addition to the same supplements the control group received. Results: There was no significant difference (*p* = 0.06) between Ct-values of the two groups before the regimen was started (day zero), indicating that subjects in both groups had similar viral loads. At 72 h after the regimen started, the increase in Ct-values was dramatically higher in the ivermectin than in the control group. In the ivermectin group, Ct increased from 15.13 ± 2.07 (day zero) to 30.14 ± 6.22 (day three; mean ± SD), compared to the control group, where the Ct values increased only from 14.20 ± 2.48 (day zero) to 18.96 ± 3.26 (day three; mean ± SD). Moreover, more subjects in the control group developed clinical symptoms. Three individuals (6%) required hospitalization, compared to the ivermectin group (0%). Conclusion: Ivermectin appears to be efficacious in providing clinical benefits in a randomized treatment of asymptomatic SARS-CoV-2-positive subjects, effectively resulting in fewer symptoms, lower viral load and reduced hospital admissions. However, larger-scale trials are warranted for this conclusion to be further cemented.

## 1. Introduction 

Regrettably, no medications or other therapies to combat or mitigate COVID-19 have been approved by the Food and Drug Administration (FDA) to date [1,2,3,4,5,6,7]. Mitigation strategies and supportive treatments, such as supplementary oxygen and artificial respiratory assistance, are the main modes of therapy for critical patients [8]. However, following the outbreak of SARS-CoV-2, numerous repurposed drugs, such as lopinavir/ritonavir combination, hydroxychloroquine or azithromycin, have been proposed or used in human clinical trials for the treatment of COVID-19 [7,9,10,11]. Very recently, studies suggested that ivermectin, an FDA-approved anti-parasitic agent since 1981, could inhibit SARS-CoV-2 [12].

Ivermectin is being examined in the context of treatment of several infectious diseases including Zika virus, dengue virus (DENV), yellow fever, avian influenza, porcine reproductive and respiratory syndrome and HIV Type 1, among others [13]. Ivermectin is an anthelmintic drug [14], and has been a constituent of the WHO’s List of Essential Medicines for a long time. It is a 22, 23-dihydro derivative of the macrocyclic lactone avermectin B1, and belongs to the avermectin family of mectin B. Mectin B itself is formed from macrocyclic lactones produced by the Streptomyces avermitilis bacterium. Its antiviral activity is based on the inhibition of the nuclear import of viral and host proteins by targeting importin IMPα/β1 [15]. Moreover, ivermectin acts against certain viral proteins, including non-structural protein 5 of DENV [16]. Importantly, the use of ivermectin demonstrated a clear suppression of RNA viruses such as DENV 1–4 [17], West Nile [15] and influenza [18]. The wide spectrum efficacy was assumed to be due to the dependency of several different RNA viruses on IMPα/β1 upon culminating infection [19,20]. Contextually, SARS-CoV protein experiments have demonstrated a possible function for IMP alpha/β1 throughout infection in signal-dependent nucleocytoplasmic SARS-CoV protein shutdown [21]. Moreover, the SARS-CoV attachment protein ORF6 was demonstrated to antagonize the antiviral action of the STAT1 transcription factor. In addition, DENV, which was responsive to ivermectin, shares similar symptoms as those developed by COVID-19 patients, such as fever and an itchy rash [22]. Brought together, these studies suggest that the inhibitory action of nuclear transport by ivermectin could also be successful against SARS-CoV-2 [19,23]. In vitro studies further encouraged a promising outcome for the use of ivermectin against SARS-CoV-2. For example, Vero/hSLAM cells contaminated with SARS-CoV-2 virus were subjected to serial dilutions of ivermectin [19]. The findings revealed a decrease in viral RNA of >5000, culminating in a 99.98% decrease in viral RNA within the cells. Moreover, no adverse effects were detected at any of the tested doses [24]. Indeed, very recently, it was shown that a single dose of ivermectin may stop the development of the SARS-CoV-2 in cultured cells by effectively eliminating the entire viral genome within 48 h [24].

Considering the aforementioned results, ivermectin is increasingly regarded as a possible drug to treat patients infected with SARS-CoV-2. Given the millions of lives that have been claimed by the virus and the intense wave of infections spreading throughout Lebanon, it was urgent and imperative to carry out human clinical trials on patients of COVID-19. Indeed, a recent paper called for a randomized controlled trial to validate the potential use of ivermectin in this debilitating disease [25]. For these reasons, this study aims to evaluate the efficacy of ivermectin in producing favorable clinical outcomes and decreasing the viral load among asymptomatic SARS-CoV-2-positive subjects. It is important to mention that there are many ongoing clinical trials investigating the potential benefit of using ivermectin for the management of COVID-19. In Lebanon, however, this is the first study to tackle this question.

## 2. Materials and Methods

This study was conducted between September and November 2020 and has been registered in the World Health Organization Clinical Trial Registry (ChiCTR2000033627) as a clinical trial. It aims to examine the effect of a single dose of ivermectin on asymptomatic SARS-CoV-2-positive subjects. This study involved 100 asymptomatic subjects who had a PCR screening test 5 days after having come in contact with suspected or positive cases of SARS-CoV2. This was done as we do not have the history of their contact exposure and the period of 5 days is recommended in Lebanon to avoid false negatives in the PCR results. The PCR testing was carried out at one designated hospital, which adheres to the instructions of the Lebanese Ministry of Public Health and the guidelines of the World Health Organization.

The SARS-CoV-2 R-GENE^®^ kit was used according to the manufacturer’s protocol (bioMérieux, Craponne, France). Briefly, the amplification program used included reverse transcription at 50 °C for 5 min, followed by Taq polymerase activation (95 °C, 15 min), then amplification (denaturation (95 °C, 10 s), annealing (60 °C, 40 s), and elongation (72 °C, 25 s), all for a total of 45 cycles.

All subjects selected were taking Zinc (30–50 mg/day) and Vitamin C (500 mg BID, twice daily) supplements as a recommended prophylactic strategy in Lebanon; these values are well within the accepted regimen [26,27] and are being used by other clinical trials such as NCT04342728. Our trial consisted of a 10-day follow-up, case-controlled approach and was conducted under the approval of the Institutional Review Board (IRB) of Rayak Hospital (accredited by the Ministry of Public Health, Lebanon). A written consent, assuring participating subjects that all information would be confidential and used only for research purposes, was obtained. Selection criteria included adult subjects whose weight is ≥45 kg and are SARS-CoV-2-positive based on a PCR result showing a Ct value below 20. Additional information about demographics and medical history were documented during randomization. Exclusion criteria included lactating or pregnant ladies, history of allergy to a component of the used medication, end-stage kidney or liver diseases, pulmonary fibrosis, advanced COPD, heart failure NYHA class IV, and recent cardiac intervention (less than two months). Based on the daily PCR results provided to the research teams, the subjects were contacted by phone and informed about the study that is based on the repositioning of a previously available drug, its side effects and potential benefits, such as reduction of potential symptoms and decreased viral load and quarantine duration. Participation was strictly voluntary and the right of withdrawal at any time of enrolment was explained and documented in the written consent.

In order to reach a balanced homogenous sample, the subjects were randomized (using stratified randomization) according to their characteristics of age, gender, marital status, and co-existing medical conditions and chronic diseases. After that, the subjects within each stratum were enlisted into separate digitally generated randomization schedules and assigned randomly to either the control or ivermectin group. Subjects in the treatment group were divided into cases who received a single dose of the drug. Subjects with body weights of 45–64 kg, 65–84 kg, or above 85 kg received (PO) 9 mg, 12 mg, or 150 μg/kg body weight of ivermectin, respectively. This dosing regimen was based on the standard approved dose as well as the safety profile of ivermectin, where doses up to 400 µg/kg are known to not exacerbate any adverse effects of ivermectin [28,29,30]. Indeed, previous evidence shows that the utilization of the normal therapeutic dosage of ivermectin (9 mg once daily) in severely afflicted COVID-19 patients was correlated with several instances of accelerated clinical improvement; clinical trials assessing its efficacy in this respect are pending [28]. This is also supported in a very recent publication showing the effectiveness of the use of similar dosing on the clinical outcomes of COVID-19 patients [29]. In addition, treatment group patients received zinc and vitamin C supplements, similar to the control group (Figure 1).

All subjects received the corresponding dose of ivermectin the day after PCR results. All participants had normal baseline creatinine and liver function tests. To collect the needed data, the participants were contacted by phone at their preferred time by the designated physician on a daily basis to assess any appearance of COVID-19-related signs and symptoms, and to evaluate the need of a specialized health care provider referral. The physician who contacted the patients for follow up did not know if they were assigned to the ivermectin or control group. All subjects underwent a second PCR test after 72 h of randomization. The viral presence between both groups was measured using cycle threshold indicator (Ct-values). Ct-values provide a relative measure of the amount of virus in the sample, but not the actual amount of virus present. The Ct-value can potentially provide a measure of copy number, if different standards of known amounts are included in the same PCR experiment and tested in parallel. The Ct-value associated with a given quantity of the standard is then used to determine by extrapolation the quantity of virus in the sample from the Ct-value produced during the test. A Ct-value of 30 and higher was considered indicative of insignificant viral remnants or a non-viable virus [31].

The official documents of the PCR and Ct-value results were photographed and sent to the designated physician for data collection and follow up. For sample size and power of the study, a prior statistical power analysis using GPower 3.1.9.2 software (Heinrich-Heine-Universität, Düsseldorf, Germany) revealed that the sample size *n* = 100 was enough to attain a statistical power of at least 80% with alpha error of 5%, balanced on each side, and effect size set to 0.56.

Statistical analysis was performed using SPSS (IBM Corp., Released 2013, SPSS Statistics for Windows Version 22.0, Armonk, NY, USA), where the plan of data analysis has entailed the expression of categorical and continuous variables as frequencies and percentages, and mean ± standard deviation, respectively. Normality was assessed using the Kolmogorov–Simonov test. Descriptive analysis was carried out to evaluate the characteristics of the subjects, while inferential statistics and namely a Mann–Whitney U test was carried out to test the homogeneity of the sample before carrying on with the intervention as well as test the differences in the outcomes after the intervention. The Mann–Whitney U test was also performed to test the difference in Ct-values between the control and ivermectin group. The analysis plan also entailed carrying out a regression analysis to identify the predictors of higher Ct-values. The Chi-squared test was used to assess any significant association between the categorical variables. The level of significance was set at *p* < 0.05 for all statistical analyses. An additional test was performed to detect outliers. Finally, to compare improvement between groups, effect size for Ct-value was calculated. The effect size (d) of different parameters (day zero vs. day three) was calculated using the equation $\;d=\frac{\mu_{1}-\mu_{2}}{S_{p}}$, where d is Cohen’s effect size; $\mu_{1}$,$\;\mu_{2}$ are pre- and post-intervention means, and $S_{p}$ is the pooled estimate of variance calculated as follows: $S_{p}=\sqrt{\frac{\left(n_{1}-1\right)S_{1}^{2}+\left(n_{2}-1\right)S_{2}^{2}}{n_{1}+n_{2}-2}}$, where $\;n_{1}$, $\;n_{2}$ are pre- and post-intervention sample sizes and $\;S_{1}$, $S_{2}\;$ are pre- and post-intervention standard deviations.

## 3. Results

### 3.1. Subjects

Of the 152 positive cases who were present at the time of the study and have been evaluated for their suitability to meet the inclusion criteria of the study, 100 age-matched patients were randomized whereby 50 subjects were included in the control group receiving prophylactic supplements for COVID-19. The other 50 patients were assigned to the experimental group receiving the same supplements, in addition to ivermectin as a potential treatment for COVID-19. Both groups had equal distribution of males and females and had a comparable age distribution, with the mean age being 31.58 ± 7.68 or 31.78 ± 7.85 in the control or ivermectin groups, respectively (Table 1). Most subjects were previously healthy, although some had one or two pre-existing conditions at the time of enrolling in the study. These conditions were roughly equally distributed among Type 2 diabetes, hypertension, dyslipidemia, neuropathy and vitamin D deficiency in both control and treatment groups. However, and rather interestingly, some subjects that were randomized into the treatment group uniquely presented with hyperuricemia, though this was not a statistically significant difference (Table 1). A Chi-squared test was carried out and the results showed no significant association between the two study groups according to subject characteristics (Table 1).

### 3.2. Clinical and Viral Outcomes

The average blood pressure was 125/71 mm Hg or 124/70 mm Hg in the control or ivermectin group, respectively. All subjects had an SpO_2_ of 95% or higher. Respiratory rate ranged from 15 to 18 in both groups. The temperature range for both groups was 36.5 to 37.2 °C. Except for the three patients who were hospitalized (from the group not receiving ivermectin), no subjects had any significant changes in these parameters throughout the study period.

Inferential statistical analysis shows that subjects in the ivermectin group developed less symptoms of fever (2% vs. 22%), anosmia (6% vs. 32%), myalgia (0% vs. 18%), and loss of taste (6% vs. 24%) in comparison with the control group (*p* = 0.002, *p* = 0.001, *p* = 0.002, and *p* = 0.012, respectively). In addition, three (6%) patients receiving standard treatment in the control group needed hospitalization throughout the process, while none of the patients receiving ivermectin needed to be hospitalized (*p* = 0.079).

A Mann–Whitney U test was carried out to determine the homogeneity of the sample. There was no significant difference (*p* = 0.058) between Ct-values of the two groups before the regimen was started (day zero), indicating that subjects in both groups had similar viral load. Seventy-two hours after the regimen started, ivermectin significantly increased the Ct-value from 15.13 ± 2.07 to 30.14 ± 6.22 (*p* < 0.001). In comparison, the Ct-value for the control group increased from 14.20 ± 2.48 to 18.96 ± 3.26 (*p* < 0.001) (Figure 2, Table 2). The effect size for the control group and the experimental group was 1.64 and 3.24, respectively. This strongly indicates an increase (~ double) in the Ct-value in the experimental group. This leads to a ~2200-fold difference between the ivermectin and control groups at 72 h (Ct 30 vs. 18.9).

To determine if a role for gender is existent in the clinical outcome, we compared the Ct values obtained across males and females. Table 3 shows that there is no significant difference between males and females regarding the progression of Ct-value (Table 3).

The results show a significant increase in the Ct-value in the experimental group for males and females following ivermectin treatment (*p* < 0.001) (Table 4).

A multiple regression was run to predict Ct-value after 72 h of treatment from age, gender, and groups (control vs. ivermectin). These variables statistically predict Ct-value after 72 h of treatment, F(3,96) = 41.540, *p* < 0.001, R^2^ = 0.565. According to Table 5, ivermectin is a predictor of higher Ct-value (*p* < 0.001). Furthermore, neither gender nor age were predictors of higher Ct-value (*p* > 0.05).

## 4. Discussion

The world is racing to find a treatment for COVID-19. The existing routine treatment for patients with COVID-19 is symptomatic rather than curative. In some practice, steroid medication for severe/critical cases, or large doses of vitamin D3, vitamin C and zinc for mild–moderate cases, have been initiated [32,33,34]. The effects of zinc could be attributed to its potential ability to inhibit Mpro of SARS-CoV-2, as has been very recently suggested [35]. As of yet, there is no standard treatment for SARS-CoV-2. Clinical trials have been revolving around drug upcycling. For incurable diseases such as COVID-19, the use of FDA-approved and effective antiviral or immunomodulatory drugs is clinically supported. Many COVID-19 patients progressing to serious illness develop elevated SARS-CoV-2 viral load and an exaggerated immune response [36,37].

In order to ensure the safety of patients, lowering the viral load and muffling both the immune response and inflammatory cytokines are important factors to be considered. Ivermectin has a documented safety profile, and is authorized by the FDA for parasitic indications [38]. Recent in vitro studies have demonstrated that ivermectin might have antiviral activity against SARS-CoV-2, where a single dose might be able to control viral replication within 24–48 h. This has been linked to the inhibition of IMPα/β1-mediated nuclear import of viral proteins [15].

Here, in this study, we evaluated the effects of ivermectin on the clinical outcomes of SARS-CoV-2-infected patients and the Ct-value progression. Our results showed that the use of ivermectin in asymptomatic SARS-CoV-2-positive subjects was significantly associated with a dramatic increase in the Ct-value.

Perhaps most notable of the findings is the time needed to clear subjects of the viral load. This has become increasingly critical as the world spins into higher rates of infection and death, especially in light of new and reportedly mutated viral strains. In our study, subjects who received ivermectin more rapidly became SARS-CoV-2-negative. Furthermore, our results were also supported by recent research demonstrating that fast virological clearing caused by ivermectin was detected, which argues in support of the therapeutic effectiveness of the medication against SARS-CoV-2. Such a quick clearance of SARS-CoV-2 (a median of 4 days) is much shorter than the median period (20 days) of viral shedding in subjects with COVID-19 who do not receive the drug. This may strongly suggest that ivermectin can restrict viral dissemination [15]. A very recent study involving 72 hospitalized adult patients with mild symptoms showed that ivermectin is safe and effective in producing earlier recovery [29]. A previous study also found results that came in line with our findings, where it was reported that ivermectin lowers mortality rates of SARS-CoV-2-infected patients more than any standard treatment or hydroxychloroquine, even among patients with pulmonary comorbidities [39]. However, in this study, the authors only focused on mortality, rather than clearance of the virus, and other clinical symptoms that we have reported here. Interestingly, the authors themselves called for randomized controlled studies. Our study supports the use of ivermectin in the management of SARS-CoV2-infected subjects, though more extensive research and large-scale trials are critically warranted. This becomes increasingly important as the vaccine is not yet available for all countries, and the rate of infections is dramatically increasing.

From a pharmacokinetic perspective, it is notable that the amount of ivermectin in lung parenchyma of rats was reported to be two-fold higher than those in blood [40]. The antiviral and anti-inflammatory effects on lung tissue were also apparent. These results further support the argument that in addition to being used as an antiviral agent, ivermectin is a potent immunomodulator. Moreover, our results are also in line with a similar study we performed in Iraq, which found that in the randomized COVID-19 cases, ivermectin decreased the average time for recovery from 17.9 to 10.61 days (unpublished data). Similarly, ivermectin–doxycycline decreased the average period to rehabilitation from 13.66 to just 6.34 days for mild intermediate patients, with time improvement to 7.32 days. Nevertheless, in critical patients, ivermectin–doxycycline shortened the average recovery duration by just 4 days, from 24 to 20 days [41]. It is important to note here that while our approach was different, similar findings have been reported by a recent paper, whereby patients treated with ivermectin tend to have lower viral loads and IgG titers, indicative of a milder disease, as well as a clinical benefit to many COVID-19 symptoms [42].

## 5. Conclusions and Recommendations

This paper provides promising evidence supporting the use of ivermectin as a medical treatment for COVID-19. Here, we indeed established ivermectin’s clinical efficiency in reducing the incidence of severe symptomatology and in significantly reducing viral loads. A limitation of this study would be that the compliance of the patients has not been monitored and drug plasma concentration was not measured. Moreover, we did not collect follow-up information from patients on the potential use of self-medications that might have interfered with the outcomes. It is also worth mentioning that these subjects undertook the PCR test not because they had any symptoms but rather because they had a suspicion that they may have come in contact with a SARS-CoV-2-positive subject. Typically, in Lebanon, subjects who come in contact with a suspected SARS-CoV-2-positive individual refer to the laboratory for a PCR test within 4–7 days. Hence, while it is impossible to confirm when exactly they may have had exposure to the virus, the test is usually taken within the early phase of the potential infection.

Because of all these limitations, we are in the process of recruiting a much larger pool of SARS-CoV-2 patients to arrive at a stronger conclusion. In this or any other higher-scale study, blood samples to review complete blood count and inflammatory parameters—as well as correlate their values with the response and liver tests—would be warranted, especially to determine tolerance and longer-term effects on the patients. Nonetheless, with the significant findings herein, we thought this pilot study may help others consider the repurposing of ivermectin, alone or in combination with other drugs, for the debilitating effects of COVID-19. Therefore, this study supports previous research indicating that ivermectin may be useful in the management of COVID-19.

## Figures and Tables

**Figure 1:** Flow chart of participant enrollment and randomization.

**Figure 2:** Bar chart showing threshold cycle (Ct-value) progression from baseline to 72 h after standard treatment in the control group. Descriptive analysis and comparison of means showed minimal increase in the Ct-value among participants in the control group.

**Table 1:** Participant Characteristics.

		Control Group	Ivermectin	*p*-Value
Gender	Male	25 (50%)	25 (50%)	1.000
	Female	25 (50%)	25 (50%)	
Marital Status	Single	20 (40%)	29 (58%)	0.072
	Married	30 (60%)	21 (42%)	
Age (mean ± SD)		31.58 ± 7.68	31.78 ± 7.85	0.830
Height (mean ± SD)		172.54 ± 7.84	172.72 ± 14.39	0.098
Weight (mean ± SD)		72.52 ± 17.28	78.00 ± 16.32	0.231
Co-existing Conditions				
	Diabetes mellitus	3 (6%)	3 (6%)	1.000
	Hypertension	4 (8%)	4 (8%)	1.000
	Dyslipidemia	3 (6%)	3 (6%)	1.000
	Neuropathy	4 (8%)	4 (8%)	1.000
	Vit. D deficiency	4 (8%)	4 (8%)	1.000
	Hyperuricemia	0 (0%)	3 (6%)	0.079

**Table 2:** Clinical Presentation of Subjects after 72 h of Treatment.

	Control		Ivermectin		*p*-Value
	N	%	N	%	
Fever	11	22	1	2	0.002
Cough	5	10	2	4	0.240
Runny Nose	2	4	1	2	0.558
Headache	5	10	2	4	0.240
Anosmia	16	32	3	6	0.001
Myalgia	9	18	0	0	0.002
Loss of Taste	12	24	3	6	0.012
Fatigue	3	6	0	0	0.079
Dizziness	2	4	0	0	0.153
Hospitalization	3	6	0	0	0.079
Ct-value; Day zero	14.20 ± 2.48		15.13 ± 2.07		0.058
Ct-value; Day three	18.96 ± 3.26		30.14 ± 6.22		<0.001

**Table 3:** Differences in Ct-value According to Gender.

	Female		Male		
	Mean	SD	Mean	SD	*p*-Value
Ct-value (Day zero)	14.93	2.71	15.27	2.87	0.544
Ct-value (Day three)	24.39	7.10	24.72	7.93	0.828

**Table 4:** Differences in Ct-value Between the Study Groups According to Gender.

		Control	Ivermectin	*p*-Value
Females	Ct-value (Day zero)	14.40 ± 2.56	15.46 ± 2.81	0.375
	Ct-value (Day three)	18.76 ± 3.36	30.02 ± 5.06	<0.001
Males	Ct-value (Day zero)	13.99 ± 2.42	15.47 ± 1.87	0.058
	Ct-value (Day three)	19.16 ± 3.22	30.27 ± 7.32	<0.001

**Table 5:** Ivermectin Predictor of Higher Ct-value after 72 h of Treatment with Ivermectin.

	Coefficients	Standard Error	*p*-Value
Age	0.03	0.06	0.655
Gender	−0.35	1.00	0.731
Group	11.18	1.00	<0.001

## Data Availability

All data are available with researchers at the Lebanese University, Faculty of Public Health IV, Zahle. Lebanon.
